The article "The Effect of Gastric Acid on the Surface Properties of Different Universal Composites: A SEM Study" was published in 2022. Journal: Scanning.

# The Effect of Gastric Acid on the Surface Properties of Different Universal Composites: A SEM Study

**DOI:** 10.1155/2022/9217802

**Published:** 2022-12-28

**Authors:** Cemile Kedici Alp, Ceyda Gündogdu, Cansu Dağdelen Ahısha

**Affiliations:** ^1^Faculty of Dentistry, Department of Restorative Dentistry, Gazi University, Emek, Ankara, Turkey; ^2^Faculty of Dentistry, Department of Restorative Dentistry, İstanbul Medipol University, Bagcılar, Istanbul, Turkey

## Abstract

The aim of this study is to compare surface roughness and microhardness changes of three monochromatic (Omnichroma, Vittra Unique, and Charisma Diamond One) and three universal shade (Neo Spectra ST, G*-*ænial A'CHORD, and Nova Compo C) resin composites after exposure to simulated gastric acid. A total of 144 disc-shaped specimens (24 discs of each composite resin) were prepared using plexiglass molds (*R* = 5 mm × *h* = 2 mm) for evaluation from each material. Specimens of each material were divided into two main groups for the evaluation of the microhardness and surface roughness and also two subgroups for 7- and 14-day exposures to simulated gastric acid. Initial microhardness and surface roughness measurements of all samples were measured before immersion (T1) followed by exposing the samples to simulated gastric acid for 7 days (T2) and 14 days (T3), and then, the microhardness and roughness measurements were repeated. Randomly selected specimens of each material for each of the time intervals (T1, T2, and T3) were evaluated with scanning electron microscopy (SEM). One-way ANOVA revealed that the surface roughness and hardness values of all tested composite resin restorative materials show no statistically significant difference for the initial (T1) value (*p* > 0.05). Regarding the 7^th^ day (T2) and 14^th^ day (T3) surface roughness and microhardness value of all composites, there are statistically significant differences between the groups (*p* < 0.05), while there was no statistically significant difference between the surface hardness reduction percentage between the time intervals (*p* > 0.05). As a result of this *in vitro* study, increase in surface roughness and decrease in microhardness of the tested universal composite materials when exposed to simulated gastric acid were statistically significant.

## 1. Introduction

Development of the adhesive techniques is increasingly trending towards more conservative and aesthetic rehabilitations for the resin composites that are used for anterior and posterior restorations due to the known different effects of amalgam. The main requirement of anterior restoration is to provide excellent color harmony with the tooth and surrounding tissues after the application. Therefore, monochromatic resin composites are developed to eliminate the process of shade selection [1]. These composites contain no dyes or pigments, and color matching ability is dependent on the special structure of the material which reflects the color of the surrounding dental structures [2].

The article "The Effect of Gastric Acid on the Surface Properties of Different Universal Composites: A SEM Study" was published in 2022. Journal: Scanning.

Restorative materials are regularly exposed to the dynamic challenges in the oral cavity such as oral masticatory forces and changes on pH and temperature [3]. In order to avoid the negative effects of all these challenges on teeth and restorations, the restorative materials should possess ideal properties of strength and durability in the intraoral complex.

Salivary pH changes extrinsically with the diet, consumption of medications, and beverages and intrinsically with gastric acid [4]. The human average intraoral pH is around 7.4 while that of gastric acid is between 1-1.5 [5]. Therefore, gastric acid has an impact on decreasing the salivary pH while buffering the capacity of saliva that protects teeth erosion from an acid attack [4]. However, the determined buffering capacity of saliva is not sufficient in patient who suffers from gastroesophageal reflux disease (GERD) [6].

Gastroesophageal reflux is caused by the reflux of the gastric contents into the oesophagus or beyond into the oral cavity [7]. Studies have found a relationship between GERD-induced reflux and dental erosion in children and adults [8–10]. As a result of vomiting, regurgitation, and GERD, the pH levels of saliva drop below 5.5, which is the critical demineralization point of enamel and can lead to dental erosion followed by loss of tooth surfaces without a bacterial involvement [6]. As a consequence of the innovations in adhesive materials, it has become possible to restore tooth structure aesthetically which is changed by dental erosion in a minimal invasive approach with resin composites [11].

The surface properties of the composite resins are directly related to aesthetic and mechanical properties of the restoration. Reduced surface microhardness results in the material being prone to scratching and roughness while also causing loss of gloss and discoloration and plaque accumulation following the bacterial adhesion [12, 13]. While the surface roughness is intrinsically related to the filler size, shape, type, and polymer matrix of the materials, it is also extrinsically related to the conditions such as acidity of foods, temperature change, and occlusal forces [14, 15]. Roughened surfaces cause more plaque accumulation than smoother surfaces and also show wear and staining on the material's surface [16].

As the material's mechanical and physical properties may be weakened by the chemicals, the material must have sufficient hardness for the longevity and success of the restoration. Although resin composites are more stable due to the formulation of the material and their filler morphology in an acidic environment, decrease in the pH values in the intraoral cavity may have negative effects on the mechanical properties of composite restorations as well [17]. Acidic pH solutions cause hydrolysis of methacrylate ester bonds in the resin matrix of polymer-based materials, causing rapid degradation of the polymer network and a decrease in the strength of the physical properties of the material such as roughness and microhardness [18, 19].

The article "The Effect of Gastric Acid on the Surface Properties of Different Universal Composites: A SEM Study" was published in 2022. Journal: Scanning.

The purpose of the present *in vitro* study was to compare surface roughness and microhardness changes of the six different universal resin composites after exposure to simulated gastric acid by using profilometer and Vickers microhardness tester machine to determine the surface changes using scanning electron microscopy (SEM).

The null hypotheses were (1) the simulated gastric acid does not affect the microhardness and roughness of the different restorative materials. (2) The time of immersion in simulated gastric acid does not affect the microhardness and roughness of the different restorative materials.

## 2. Material and Method

In this study, the effect of gastric acid on the six different composites that are categorized as monochromatic and universal shade was investigated. A sample size of the study determined by the G^∗^Power ver. 3.1.9.4 (Prof. Dr. Franz Faupel, Uni Kiel, Germany) software with an error probability of *a* = 0.05, an effect size *d* = 1.87, and 95% power.

Three monochromatic (Omnichroma, Vittra Unique, and Charisma Diamond One) and three universal shade (Neo Spectra ST, G-ænial A'CHORD, and Nova Compo C) resin composites were selected for this study. The technical properties of the composite resin restorative materials used in this study are shown in Table 1. A total of 144 disc-shaped specimens (24 discs of each composite resin) of 5 mm in diameter and 2 mm thickness were prepared using standardized plexiglass molds for surface roughness and microhardness evaluations from each material. The composite resins were condensed as a single increment into the mold, and then, glass slide and Mylar strips were positioned with light pressure on both surfaces to remove the excess material. Each specimen was then photopolymerized using a LED curing unit (D-Light Pro, GC, Leuven, Belgium) with a wavelength of 430-480 nm and a light intensity of 1.200 mW/cm^2^ according to the manufacturer's instructions. The light intensity of the curing unit was checked regularly for every five exposures using a light radiometer (LED Radiometer, Kerr, Orange, CA, USA). After the light application, specimens were stored in distilled water at 37°C for 24 hours in a dark environment because of postpolymerization. Samples were prepared and tested in the same laboratory by the same operator using the same equipment within short intervals of time to ensure standardization. The bottom surfaces of the specimens were marked with a scalpel.

The article "The Effect of Gastric Acid on the Surface Properties of Different Universal Composites: A SEM Study" was published in 2022. Journal: Scanning.

Polishing procedure was performed with Shofu (Super-Snap, Shofu Inc., Japan) coarse, medium, fine, and superfine aluminum oxide abrasive discs using a low-speed dental handpiece (15,000 RPM). After each disc is used for the application, the specimens were rinsed for 10 seconds and dried with light air for 5 seconds to remove the polishing debris. The simulated gastric acid was pepsin-free and consisted of 0.06 M and 0.113% HCl (pH 1.2 ± 0.2) acid solution in distilled water. During the study, gastric acid solution was freshly formulated daily.

Specimens of each material were divided into two main groups for the evaluation of the microhardness and surface roughness and also two subgroups (*n* = 6) as 7-day and 14-day exposures to simulated gastric acid.

Initial microhardness and surface roughness measurements of all samples were measured before immersion with gastric acid from the top surfaces. First measurement (T1) of surface roughness was assessed using stylus profilometer (Surftest SJ-301; Mitutoyo, Illinois, USA) with an area of 100∗100 *μ*m^2^. The Vickers hardness number (VHN) (kg/mm^2^) of composite resin materials was determined with a Vickers microhardness tester (HMV-2; Shimadzu, Tokyo, Japan) under 490 *μ*N load for 15 seconds. The measurements were repeated five times at randomly selected five different points by rotating the specimen around its center in a clockwise direction, and the average values were calculated.

After the initial measurements were completed, the samples were exposed to 18 hours of simulated gastric acid solution and 6 hours of distilled water per day for 7-day (T2) and 14-day (T3) time intervals, and then, the microhardness and roughness measurements were repeated. Composite specimens were put into the glass Petri dish at 37°C for 14 days in 100% humidity in simulated gastric acid for 18 hours/day followed by 6 hours/day in distilled water [20, 21]. Before the measurements, the specimens were washed in distilled water and blotted dried with absorbent paper.

Randomly selected specimens of each material for each of the time intervals (T1, T2, and T3) were coated with gold (Leica EM ACE200, Leica Microsystems, Washington DC, USA) and evaluated with scanning electron microscopy (Hitachi SU5000 FE-SEM). The entire surface of these specimens was scanned, and photographs were obtained at 10000x magnifications from the areas showing surface structure by high vacuum SEM, operating at 1 Torr pressure and 10 kV.

The article "The Effect of Gastric Acid on the Surface Properties of Different Universal Composites: A SEM Study" was published in 2022. Journal: Scanning.

## 3. Statistical Analysis

The data was analyzed with software SPSS software package version 22.0.0.0 (IBM Corp., ILL, Chicago). According to the Shapiro-Wilk test, surface roughness and microhardness data sets were normally distributed where significance *p* value (0.05) indicates the normality assumption. Analyses of variance (ANOVA) were used to compare the means of the surface roughness and hardness and surface hardness reduction percentage (HR%). The interactions and multiple comparisons were performed using a post hoc Tukey's test. *p* values less than 0.05 were considered to be statistically significant in all tests.

## 4. Results

The surface roughness mean values for the resin composites after each time intervals are shown in Table 2. Regarding the 7^th^ day (T2) and 14^th^ day (T3) surface roughness value of monochromatic and universal shade composites, there is a significant difference between the groups (*p* < 0.05).

Surface roughness of monochromatic composites (Omnichroma, Vittra Unique, and Charisma Diamond One) was analyzed; then, Tukey's post hoc test ascertained that Vittra Unique composite's surface roughness value was significantly lower than the Omnichroma and Charisma Diamond One groups. In addition, the Charisma Diamond One group showed significantly higher surface roughness value than the Omnichroma and Vittra Unique groups after 14 days (T3) of gastric acid treatment (*p* < 0.05).

The surface roughness of the universal shade composites (Nova Compo C, G-ænial A'CHORD, and Neo Spectra ST) was examined, and the Tukey's post hoc test determined that in both time intervals (T2 and T3), surface roughness value of the Nova Compo C groups was significantly higher (*p* < 0.05).

When the 7^th^ day and 14^th^ day microhardness measurement values were compared with all the other groups, the difference was found to be statistically different (*p* < 0.05). When the microhardness of monochromatic resin composite groups was examined, the Omnichroma groups were statistically harder than the Vittra Unique and Charisma Diamond One groups in 7^th^ (T2) and 14^th^ (T3) time intervals (*p* < 0.05) (Tables 3 and 4).

The average microhardness values of the resin composites after each time interval are shown in Table 3. The surface microhardness values of the Nova Compo C group were significantly lower than the Neo Spectra ST and G-ænial A'CHORD groups in the 7^th^ (T2) and 14^th^ (T3) time intervals (*p* < 0.05).

The article "The Effect of Gastric Acid on the Surface Properties of Different Universal Composites: A SEM Study" was published in 2022. Journal: Scanning.

The impact of the simulated gastric acid on the roughness of the composite resin samples was analyzed with the Friedman test of difference, and there was a significant difference among the initial (T1) surface roughness and microhardness on the 7^th^ (T2) and 14^th^ (T3) days in all tested groups (*p* < 0.05). Regardless of the color feature, the roughness values of the samples in all groups showed statistically higher values compared to the initial measurements, while a decrease was observed in the microhardness values with the effect of gastric acid (*p* < 0.05).

When the surface hardness ratios were examined, no statistically significant difference was observed between the hardness reduction percentages of the materials between the different time intervals and different brands (*p* > 0.05).

In SEM evaluation, the surface changes are shown at Figure 1 when the composites were immersed in gastric acid for 7th days and 14th days.

Although the exposure of the samples to an acidic solution significantly increases all recorded Ra values, SEM micrographs show that the Omnichroma groups can provide durability and showed more stable surface features under gastric acid challenges when it was compared with initial time (T1) image (Figure 1(a)).

When the Charisma Diamond One and Vittra Unique groups are examined, changes in surface textures at 7- and 14-day time intervals can be observed as pores and cracks in SEM images (Figures 1(d)–1(i)). 7-day and 14-day SEM images were examined, and it can be observed that the pores on the surface of the Neo Spectra increased and deepened over time (Figures 1 and 2).

## 5. Discussion

In the present study, composite resin specimens were stored in the simulated gastric acid solutions to evaluate the effect of low pH on the microhardness and surface roughness of six different universal resin composites for 7 days (T1) and 14 days (T2). The results showed that the surface roughness and microhardness of composite resins were affected by the chemical attack of simulated gastric acid. Hence, the first null hypothesis that the simulated gastric acid does not affect with microhardness and roughness of different restorative materials was rejected. The surface roughness and the surface microharness values were decreased over the time in the simulated gastric acid. Therefore, the second null hypothesis of the present study was rejected. These findings can be supported by SEM images confirming similar amount of filler surface change after 7-day and 14-day immersions with simulated gastric acid.

Gastric acid can cause demineralization in dental hard tissues and may also dissolve resin matrix of composites during reflux due to its low pH varying between 1-1.5 [22]. In a systematic review, the median prevalence of dental erosion in GERD patients was calculated to be 24% (range between 5-47.5%), where it was 17% (range between 21-83%) of patients with dental erosion who have gastroesophageal reflux [23].

The article "The Effect of Gastric Acid on the Surface Properties of Different Universal Composites: A SEM Study" was published in 2022. Journal: Scanning.

The *in vitro* simulation method of the exposure of gastric acid onto the intraoral complex was not established, and some studies planned different immersion times from 1 day to 1 month. Cengiz et al. used gastric acid solution (pH = 1.2) for 24 hours at 37°C to simulate worst-case scenario of patient with reflux attacks [24]. Another study reported that the 6-hour and 18-hour test periods represent 2 and 8 years approximately [25]. Unal et al. and Guler and Unal determined that storing composite samples *in vitro* for 14 days in gastric acid is equivalent to 13 years of intraoral condition [20, 21]. In the present study, 126 hours (7 days) and 252 hours (14 days) test periods were used to obtain a reasonable immersion time that represents intraoral environment.

Resin composites are composed of the monomers and the inorganic filler particles such as quartz, zirconia, borosilicate, and silica [26]. The survival of resin composite restoration is directly related to the biodegradation resistance during the chemical attacks. Salivary enzymes, cariogenic biofilm, acidic foods, and gastric acids soften the resin matrix and may cause an increase in roughness and a decrease in microhardness as a result of chemical degradation [27]. Many factors such as the structural properties of the filler particles (size, type, and distribution), organic matrix, and resin-filler coupling agents are related to the degradation behavior of the restorative material [28].

It is reported that the critical surface roughness that causes bacterial colonization on the restorative material is 0.2 *μ*m. On average, tongue may distinguish roughness value when it is more than 0.5 *μ*m [16, 29]. Attar reported that if the surface roughness value is less than 1 *μ*m, it indicates an optically smooth restoration surface [30]. Similar to our results, literature shows that the exposure of the resin composites to gastric acid for 7 and 14 days results in increased surface roughness [20, 31].

Another finding of the present study was that all of the composite resins presented surface changes after being exposed to gastric acid. The SEM analysis showed several protruding particles, voids, and cracks in all specimens analyzed regardless of the time of exposure as a result of chemical erosion (Figures 1 and 2).

Consistent with surface roughness values, the results of SEM images show that the surface texture of the Charisma Diamond One and Nova Comp C groups was rougher than the other tested composite groups. This result can be explained by the differences in the monomer structure in addition to the fact that the composite materials have different filler particle size and amount. Nova Comp C contains ULS (ultralow shrinkage) monomer.

The article "The Effect of Gastric Acid on the Surface Properties of Different Universal Composites: A SEM Study" was published in 2022. Journal: Scanning.

Dental resin composites are mainly composed of organic resins, inorganic fillers, and coupling agents, and their mechanical properties are produced by the modification of inorganic filler particles [32]. Particle size of the filler has an impact on the surface roughness. Fillers with finer particle sizes in the structure of the material lead to a reduced interparticle gap and matrix which result in a more stable and wear-resistant structure [33]. The shape and size of the resin composite fillers determine the surface properties of restorations. This is because when the filler particles are removed from the surface, they leave small or large defects, depending on the size [34]. In all tested composites, the greatest surface roughness change can be observed in the first seven-day period. In addition, among the tested materials, the highest roughness was observed in Charisma Diamond One and Nova Comp C after 7 days of exposure to gastric acid. The particle size of the materials evaluated in the study was between 0.2-20 *μ*m, and the roughness was significant in the groups with higher particle size (Charisma Diamond One and Nova Compo C), similar to the studies [28, 35, 36].

The matrix/filler interface of resin composites display high sensitivity to sorption. The absorbed water may cause the degradation due to breakage of the chemical structure of the resin composites [37]. The gastric acid with high concentration of protonated protons (H^+^) accelerates the sorption process, and exposure of the polymer-based restorative materials into the low pH solutions causes hydrolysis of ester bonds from dimethacrylate monomers (TEGDMA, Bis-GMA, and UDMA) that are present in the organic matrix [38]. As a result of this process, formation of alcohol and carboxylic acid molecules causes degradation of the resin composite, weakening the physical properties of the materials [39]. Cilli et al. investigated the effect of the filler particles on surface roughness after hydrolytic degradation and determined that the water diffused into the matrix structure during hydrolysis had the effect of disrupting the surface texture, especially around the silanized inorganic particle [37].

Backer et al. reported that the hydrophilic monomers such as Bis-GMA and TEGDMA also can increase rate of hydrolysis and result with roughened surface topography [25]. Although the Charisma Diamond One, Omnichroma, and Vittra Unique groups have TEGDMA-based matrix, only the Charisma Diamond One group has significantly recorded higher roughness, which can be explained by the inorganic filling structure properties of the Omnichroma and Vittra Unique groups.

The article "The Effect of Gastric Acid on the Surface Properties of Different Universal Composites: A SEM Study" was published in 2022. Journal: Scanning.

Filler particle shape impacts the surface roughness of the composite resin materials [33]. Spherical particles are mostly obtained from silica and provide a more homogeneous flow of the structural stresses compared with the irregular glass melted-based fillers [40]. Theoretically, in contrast with our study, spherical fillers are expected to show less roughness after polishing and chemical degradation than irregular fillers, but the variation of particle size may affect the surface texture of the tested materials [41].

Manufacturers in the nanotechnology sector have recently developed nanoceramics containing polycrystalline resin matrix and nanoceramic filler with high flexural strength, where the material is biocompatible, and it has satisfactory polishing and aesthetic properties [42]. Similar to our results, Jafarnia et al. compared the roughness of nanocomposites and found that the nanoceramics have the smoothest surface roughness (G*-*ænial A'CHORD and Nova Compo C) [43].

The increase in the filler volume/weight ratio in the material also increases the wear resistance against the exposed external factors and reduces the surface roughness [44]. Charisma Diamond One composite has the lowest filler ratio (65 vol%) between the composites used in this study and has the highest surface roughness between the groups. This result may be related to the low filler ratio of the resin composite.

Surface roughness can be measured by methods that include contact stylus tracing, scanning electron microscopy (SEM), laser specular reflectance, or atomic force microscopy [11]. The most common method is the contact stylus tracing which provides 2D quantitative measurements of the surface roughness [45]. Although the quality of the data obtained from the contact and noncontact methods are controversial, Paepegaey et al. compared the two methods in their study in which they measured enamel erosion and did not detect a statistical difference between the methods [46]. Qualitative evaluation of the surface texture can be measured in 3D with SEM with a morphological approach [47]. In the present study, micrographs were taken at 10000x to give specific views of the surface topography and parameters impacting the Ra values that are obtained from the profilometer.

Increased surface roughness values in T2 and T3 time intervals may be associated with the removal of heterogeneous inorganic filler particles with different sizes (5 *μ*m-20 *μ*m). Degradation caused by gastric attacks was examined in SEM images of Charisma Diamond One (Figure 1(b)).

The article "The Effect of Gastric Acid on the Surface Properties of Different Universal Composites: A SEM Study" was published in 2022. Journal: Scanning.

Mylar strips are frequently used as a matrix during the restoration process and to produce the smoothest surfaces [48]. However, since the use of strips is limited and complex in certain types especially of posterior restorations and does not fully reflect the clinic, we polished the samples with Sof-Lex polishing kit, which are aluminum oxide-impregnated discs [49].

The microhardness of the restorative material defines the fracture resistance of the structure and ensures that it maintains the original shape against exerted forces. It is also related to the wear resistance and stability of the material in the intraoral complex, which undergoes a dynamic pH change during the day. Chemical attack caused by GERD can decrease the pH that softens and increases the wear of the restorative material while causing hard dental tissues [20].

Intermatrix distances were decreased, and filler particle values are increased in order to increase the physicochemical properties of the material in the nanofilled composites [50]. Dental literature indicates that the nanofilled composites lead to improved polishing ability combined with improved hardness and abrasion resistance [51]. Similar to our results, Beun et al. investigated the microhardness of microfill, nanofill, and hybrid composites in their study and found that nanofill composites had a significantly higher microhardness [52].

When the surface hardness of the materials is examined, although statistically significant differences are detected, the ratios of hardness lost by the materials against gastric acid are the same for all tested composites in the first 7 days and the first 14 days (Table 4). This may be related to the fact that the materials we tested are current composites and have similar structural properties.

Charisma Diamond One contains tricyclodecane (TCD), a very reactive monomer aimed at reducing polymerization shrinkage with low viscosity. Contrary to our findings, Frauscher and Ilie revealed that the TCD monomer is more resistant to hydrolytic degradation than Bis-GMA and TEGDMA monomers [53]. This diversity may be due to the different methods used in the studies and the materials tested. It can be attributed that TCD monomer may be unstable in the gastric acid conditions.

Filler particles in a resin matrix enhance mechanical properties such as microhardness and surface roughness. Increased filler loading has been shown to result in increased microhardness and decreased water absorption with less surface degradation [54, 55]. Although Nova Compo C and Vittra Unique had the lowest filler ratios, all tested composites except Omnichroma and Neo Spectra showed similar microhardness values after exposure to simulated gastric acid. The better micromechanical properties of Omnichroma can be attributed to supra-nanospherical fillers and lack of Bis-GMA in organic matrix, while Neo Spectra contains neither Bis-GMA nor TEGDMA [56]. Also, the fact that Nova Compo C has the highest roughness and lowest microhardness values after exposure to gastric acid may be due to hydrolytic degradation caused by low pH.

The article "The Effect of Gastric Acid on the Surface Properties of Different Universal Composites: A SEM Study" was published in 2022. Journal: Scanning.

Dental resin composites may contain different types of metallic fillers such as barium zinc and quartz, which affect the behavior of the structure [26]. The decrease in the pH value in the environment may lead to the degradation of filler particles such as barium, quartz, and silica [57]. In addition, since barium, which is an electropositive element, reacts with water, it may undergo hydrolytic degradation and lead to a decrease in the mechanical properties of the structure [58]. Yap et al. found that barium glasses dissolve more in acidic solutions than quartz glasses, which results with the decrease in surface microhardness [28]. Nova Compo C and Charisma Diamond One samples may have been the groups with the lowest microhardness after exposure to gastric acid solutions due to the Ba filler particles they contain.

The morphology of the filler particles also affects the mechanical properties of resin composites [54]. The fact that Charisma Diamond One has the lowest hardness and highest roughness among the tested composites after exposure to simulated gastric acid can be explained by the prepolymerized filler particles in the structure which may cause the weak cross-linking between the polymer matrix and the fillers [59].

## 6. Conclusions

Within the limitations of this study, the following conclusions can be drawn:

1. Exposure to simulated gastric acid for 7 days and 14 days showed statistically significant increase in the surface roughness and decrease in microhardness of the tested composite material
2. After 7 days of exposure to gastric acid, the roughness of all materials was clinically acceptable. After 14 days, all composites were clinically acceptable except for the Nova Compo C and Charisma Diamond One groups
3. Surface roughness and microhardness depends on the type and composition of the restorative material used
4. Omnichroma composite is more stable than the other tested materials that can be attributed to its high microhardness values because of its composition

## Figures and Tables

**Figure 1:** Scanning electron microscopy (SEM) photomicrographs of the monochromatic resin composites **(**10000x**)**. Omnichroma (first line), Charisma Diamond One (second line), and Vittra Unique (third line). (a, d, g) Initial; (b, e, h) 7^th^ day gastric acid immersion; and (c, f, i) 14^th^ day gastric acid immersion.

The article "The Effect of Gastric Acid on the Surface Properties of Different Universal Composites: A SEM Study" was published in 2022. Journal: Scanning.

**Figure 2:** Scanning electron microscopy (SEM) photomicrographs of the universal shaded composites (10000x). Neo Spectra (first line), A'CHORD (second line), and Nova Comp C (third line). (a, d, g) Initial; (b, e, h) 7^th^ day gastric acid immersion; and (c, f, i) 14^th^ day gastric acid immersion.

**Table 1:** Material used in the study.

Product	Type	Shade	Filler content-filler (wt%/vol%)	Filler particle size	Manufacturer	Batch no.
Omnichroma	Nanofill resin composite	—	Supra-nanospherical fillers (260 nm spherical SiO2-ZrO2), UDMA, and TEGDMA (79 wt%/68 vol%)	2.6 *μ*m	Tokuyama, Tokyo, Japan	010E70
Charisma Diamond One	Nanohybrid resin composite	—	Advanced TCD (tricyclodecane) Matrix, BPA-free, and BrF_2_ (82 wt%/65 vol%)	5 *μ*m-20 *μ*m	Heraeus Kulzer GmbH, Hanau, Hesse, Germany	K010021
Vittra Unique	Nanohybrid resin composite	—	UDMA, TEGDMA, photoinitiator composition (APS), Zr, Si, and BPA-free (72–82 wt%/52–60 vol%)	0.2 *μ*m	FGM, Joinville, Brazil	21020
Neo Spectra	Nanohybrid resin composite	A2	Methacrilate-modified polysiloxane barium glass, and ytterbium fluoride (79%/61%)	3 *μ*m-7 *μ*m	Dentsply, North Carolina, USA	2103000019
A'CHORD	Nanohybrid/nanoceramic resin composite	A2	CERASMART, Bis-MEPP, UDMA, glass filler, and fumed silica (82 wt%/65vol %)	3 *μ*m	GC, Luzern, Switzerland	2010071
Nova Compo C	Nanohybrid/nanoceramic resin composite	A2	Barium glasses, ytterbium and prepolymer, and TEGDMA (78 wt%/nondeclared)	4 *μ*m	Imicryl, Konya, Turkey	21E795

Abbreviations: Bis-MEPP: bisphenol A ethoxylate dimethacrylate; BPA: Bisphenol A; TEGDMA: triethylene glycol dimethacrylate; UDMA: diurethane dimethacrylate.

**Table 2:** Mean and standard deviations of surface roughness parameter for all tested composite resins.

Resin composites (*n* = 6)	Initial (T1) ± Std. deviation	7^th^ day (T2) ± Std. deviation	14^th^ day (T3) ± Std. deviation	*p*
Omnichroma	0.045 ± 0.03^A^	0.320 ± 0.48^b,B^	0.329 ± 0.06^d,B^	0.009
Charisma Diamond One	0.046 ± 0.11^C^	0.478 ± 0.11^a,D^	0.536 ± 0.09^c,D^	0.009
Vittra Unique	0.047 ± 0.01^E^	0.289 ± 0.85^b,F^	0.340 ± 0.07^d,F^	0.002
Neo Spectra	0.048 ± 0.16^G^	0.224 ± 0.51^b,H^	0.273 ± 0.32^d,H^	0.003
A'CHORD	0.051 ± 0.08^J^	0.202 ± 0.60^b,I^	0.203 ± 0.65^d,I^	0.011
Nova Compo C	0.059 ± 0.16^K^	0.523 ± 0.73^a,L^	0.580 ± 0.69^c,L^	0.006

^∗^Capital letters refer to statistical groupings for each evaluated time (line), and small letters indicate significant difference in roughness parameter (column) (*p* < 0.05).

The article "The Effect of Gastric Acid on the Surface Properties of Different Universal Composites: A SEM Study" was published in 2022. Journal: Scanning.

**Table 3:** Mean and standard deviations of surface hardness parameter for all tested composite resins.

Resin composites (*n* = 6)	Initial (T1) ± Std. deviation	7^th^ day (T2) ± Std.deviation	14^th^ day (*T*3) ± Std.deviation	*p*
Omnichroma	116.583 ± 12.46^A^	103.467 ± 5.72^a,B^	98.150 ± 5.14^g,C^	0.002
Charisma Diamond One	99.53 ± 5.76^D^	90.36 ± 3.53^b,E^	84.80 ± 3.49^e,F^	0.002
Vittra Unique	99.0 ± 3.57^G^	88.90 ± 2.24^b,c,H^	85.55 ± 1.45^e,h,I^	0.002
Neo Spectra	107.63 ± 7.38^J^	99.23 ± 4.49^b,d,K^	93.00 ± 2.83^f,L^	0.002
A'CHORD	108.33 ± 12.48^M^	95.817 ± 9.99^b,N^	89.80 ± 6.83^e,O^	0.002
Nova Compo C	93.30 ± 10.60^P^	82.450 ± 9.98^b,R^	76.700 ± 6.65^e,h,S^	0.006

^∗^Capital letters refer to statistical groupings for each evaluated time (line), and small letters indicate significant difference in hardness parameter (column) (*p* < 0.05).

**Table 4:** Mean and standard deviations of surface hardness reduction ratios (HR%) after 7^th^ day (T1-T2) and after 14^th^ day (T1-T2) for all tested composite resins.

Resin composites (*n* = 6)	Initial (T1)-7^th^ day (T2) ± Std. deviation	Initial (T1)-14^th^ day (T3) ± Std. deviation
Omnichroma	10.79 ± 5.32	15.31 ± 6.10
Charisma Diamond One	9.10 ± 2.86	14, 67 ± 3.94
Vittra Unique	10.12 ± 3.48	13.49 ± 3.46
Neo Spectra	7.60 ± 4.70	13.19 ± 8.21
A'CHORD	10.50 ± 3.62	15.96 ± 4.25
Nova Compo C	11.63 ± 3.47	15.47 ± 6.02

## Data Availability

The data used to support the findings of this study are available from the corresponding author upon request.
